RETRACTED

# Enhancement of the blue photoluminescence intensity for the porous silicon with HfO_2_ filling into microcavities

**DOI:** 10.1038/srep15574

**Published:** 2015-10-27

**Authors:** Ran Jiang, Xianghao Du, Weideng Sun, Zuyin Han, Zhengran Wu

**Affiliations:** 1 School of Physics, Shandong University, Jinan 250100, China

## Abstract

With HfO_2_ filled into the microcavities of the porous single-crystal silicon, the blue photoluminescence was greatly enhanced at room temperature. On one hand, HfO_2_ contributes to the light emission with the transitions of the defect levels for oxygen vacancy. On the other hand, the special filling-into-microcavities structure of HfO_2_ leads to the presence of ferroelectricity, which greatly enhances the blue emission from porous silicon. Since both HfO_2_ and Si are highly compatible with Si-based electronic industry, combined the low-cost and convenient process, the HfO_2_-filled porous Si shows a promising application prospect.

During recent years, many materials have come to attention of researchers, using as light emitting device (LED), due to the extensive commercial demand^1^,^2^. Among them InGaN, GaAs and AlGaN are mostly popular, ascribed to the satisfactory emission intensity and mature fabrication techniques^3^. However, it is big blocks against these materials for the incompatibility with Si-based microelectronics process and the expensive cost for commercial demand. Naturally, LEDs made from Si could be released from the above problems, which is easily integrated into chips resulting translation with high speed. So far no other materials achieve perfect commercial applications as Si. However, Si is hard to show strong photoluminescence emission in a similar manner as other materials, such as InGaAs^4^, due to the indirect band gap. For this study, we present experimental results that depending on a simple wet chemical process with HfO_2_ filling into a crystal Si, strong visible blue light emission can be achieved. Considering the good compatibility of HfO_2_ dielectric with Si-based electronic industry, the integration of HfO_2_ with Si is attractive for the photoelectric application^5^,^6^. Additionally, the experimental results reported here strongly support the ferroelectric characteristic in special encapsulation for hafnium oxide, which is in highly debating recently.

## Methods

### Flow process of fabrication

Substrates were prepared with a polished single crystal Si (100) wafer, which is cut into rectangle parts in order to ensure identity of all samples. Then utilizing ethanol, acetone and deionized water, substrates were fully cleaned. Afterwards, the shadow mask full of 3 μm-size- microcavities was used for patterning on Si that was coated with the special photo resist of X AR-P 3100/10. The phtolithography was applied using UV Mask Aligner of Carl Suss MJB6. The above lithography process is to confine the wet-etching region of porous silicon after developing. The porous Si was realized using anode electrochemical corrosion method. The mixture of HF and ethanol with 1:1 volume ratio was used as corrosion liquid. After 8 min corrosion under the current density of 25 mA/cm^2^, the samples were cleaned and purged using deionized water and nitrogen, respectively. After treatment to Si, sputtering fabrication of HfO_2_ was induced in the treated Si substrate in Ar/O_2_ atmosphere with 5 mTorr pressure. This sputtering process yielded HfO_2_ films about 500 nm. The relative thick layer guarantees the sufficient filling of microcavities in porous silicon as well as the dense characteristic of sputtering. Low power was used for trying to reduce the surface damage, which readily happens due to the bombardment to the fragile structure of microcavities in Si. Afterwards, the HfO_2_ films deposited on the residual photo resist were purged via lift-off process while the filled HfO_2_ in microcavities were left. During this process, silicon surface was exposed for further photoluminescence (PL) measurement. Finally, the sample was treated with a post deposition annealing (PDA) step at 500–900 °C for 30 min in vacuum and oxygen ambient, respectively. The abovementioned fabrication process was illustrated in Fig. 1. As the process finished, the original sample surface contained microcavities filled with HfO_2_ dielectric.

RETRACTED

### Characterization with instruments

PL spectra were measured through spectrofluorophotometer (RF-540) by using 325 nm line of He-Cd laser as excitation source. The film thickness was measured by ellipsometer. Fourier transform infrared (FTIR) spectra were recorded by Bomem MB-100 spectrometer using the KBr wafer technique. Polarization hysteresis loops were measured using an aixACCT TF Analyzer 1000 measurement system. X-ray differaction (XRD) was measured by a Bruker D8 XRD system with Cu Kα radiation source.

## Results and Discussion

Figure 2 shows the PL spectra for the HfO_2_-filled PS samples which were annealed in vacuum from 500 to 900 °C, respectively. Inset shows the corresponding emission images. The visible blue emission was pronounced at 900 °C, and no emission can be observed by naked eyes below 700 °C. The patterned region in shadow mask for each sample was shown in inset, it can be found the distribution of blue emission is well consistent with the pattern region in mask, which indicates that the visible blue emission is directly related to the filling structure of HfO_2_ into microcavities of porous silicon.

RETRACTED

The PL bands of PS were most pronounced located at ~480 nm and ~740 nm^7^, which is ascribed to the Si-O emission center near surface and the surface state or quantum-limited effect (QLE)^8^,^9^, respectively. The corresponding subpeaks are present in measurements, denoted as , , respectively (‘B’, ‘R’, ‘3’ and ‘Si’, denotes the bluepeak, the redpeak, the order of subpeak and the origination of emission). It is reasonable to conclude these two subpeaks as emission from Si itself. The  subpeak shows abrupt increasing at the 700 °C, and further greatly increases at 900 °C in vacuum annealing, while this subpeak keeps nearly constant below 700 °C. This abnormal result should be ascribed to the interaction of the introduced HfO_2_ with the microcavity structure of porous silicon. The ferroelectric HfO_2_ could lead to the formation of inner electrical fields with its spontaneous polarization, which attracts the photo-generated electrons and holes moving directionally. Thus, the diffusion of carriers could be greatly limited with the recombination enhanced at the HfO_2_/Si interface region, where there is Si-O emission center due to oxidation. It is known that the diffusion of carrier into point defect is generally responsible for non-radiative recombination. Even in the PS with high quality, this non-radiative recombination is predominant. Therefore, the directional transport due to the presence of ferroelectric HfO_2_ could effectively confinesthe diffusion of carriers.

As for the ferroelectricity of HfO_2_, which is key factor responsible for the enhancement of the  subpeak as assumption above, its existence is under debate recently. It is reported that the ferroelectricity of HfO_2_ is related with the mechanical encapsulation of HfO_2_ and the dopant insertion, which leads to the distortion of HfO_2_ during crystallization and phase change^10^,^11^,^12^,^13^. The ferroelectricity in HfO_2_ films originates from the existence of the metastable and non-centrosymmetric orthorhombic phase with the space group of *P*ca2_1_ 14,15. If crystallization occurs under mechanical encapsulation, the formation of the monoclinic phase is inhibited^10^, then the orthorhombic phase that shows a distinct piezoelectric response^14^,^16^,^17^,^18^,^19^,^20^ will obtained. It is 600 ~ 700 °C for HfO_2_ films crystallized according to previous reports^21^. Generally, the orthorhombic phase was shown in final step with annealing temperature increasing followed the monoclinic and tetragonal phases. However, the encapsulation of microcavities here may catalyzes the ferroelectric phase extending to lower temperatures in nano-scale crystallites due to the surface energy effect. In this work, the pure HfO_2_ located at the surface of porous Si had been removed with the lift-off process. The preserved HfO_2_ fractions with micro&nano meters size are all isolated and embedded in microcavities. Ascribed to the entire mechanical encapsulation to HfO_2_ by the microcavities of highly porous, electrochemically etched silicon, the ferroelectric HfO_2_ phase was probably formed in our samples. As shown in diagram illustration in Fig. 3, the cavities extend irregularly into the bulk of the single-crystal Si with size ranged from nanometers to micrometers. The HfO_2_ was so well encapsulated, especially at the deep region of the microcavities.

RETRACTED

Additionally, ferroelectricity of HfO_2_ is found to exist even in thin films of less than 10 nm in thickness, which could be enhanced and modulated by various dopants, such as, Si, Al and Y etc^23^,^24^,^25^. One may argue that the ferroelectricity from pure HfO_2_ was seldom reported before. However, the HfO_2_ is probably not pure but with Si incorporation in this work, because the sputtering bombardment could carry Si into the HfO_2_ in microcavities due to the fragility and the irregular shape of Si sidewall of porous micocavity^22^, as shown in inset of Fig. 3. From the comparison in cross-sectional SEM image as shown in Fig. 3(a,b), clearly HfO_2_ coverage of the sidewalls of microcavities of porous silicon could be found. Though wet etching leads to various size of cavities from the frontside view of image, and distorts the array to some extent, good formation of microcavities is present seen in Fig. 3(c).

In order to verify the purity of HfO_2_, XPS measurement for samples after annealing was shown in Fig. 3. From the deconvolution, besides the Hf 4*f* spectra of HfO_2_, a new doublet component appears (fixed at 17.4 and 18.9 eV). It is due to the formation of Hf silicides embedded in Hf silicates from the decomposition of HfSi_*x*_O_*y*_, which has been well documented by many groups^26^. With Si adjustment, it is reasonable that HfO_2_ exhibits a ferroelectric polarization^27^. Additionally, Johannes Müller^28^ and coworkers have reported the ferroelectricity in undoped hafnium oxide very recently. Structural as well as electrical evidence for the appearance of a ferroelectric phase in pure hafnium oxide was collected with respect to film thickness and thermal budget. They present experimental proof that depending on film thickness/grain size and the adjustment of thermal budget a ferroelectric phase in HfO_2_ can be achieved without the utilization of a dopant. The demanded conditions are fitly consistent with that in this work, considering the physical fabrication method, the thickness range of HfO_2_ layer and the thermal annealing budget here. However, as shown in literature for the doped systems and as these results show for the pure oxide, both are capable of inducing ferroelectricity independently of one another. The presence of ferroelectricity in HfO_2_ which filled into the microcavities of porous Si, is a dominant reason responsible for the enlargement of original blue emission from Si. Furthermore, HfO_2_ not only help to improve the bule emission from Si, it also contributes to the blue subpeaks denoted as  and  in Fig. 2. The overall blue emission which can be seen by naked eyes is probably from the coworking of HfO_2_ and Si, which are both perfect compatible with traditional microelectronics industry process.

RETRACTED

Actually, the P-V loop present ferroelectric characteristic in measurements was obtained as shown in Fig. 4a. This observation is in agreement with the XRD measurements as shown in Fig. 4b, which showed signs of an orthorhombic phase for 700 °C annealing, as well as the temperature higher than 700 °C, such as 900 °C (data not shown). The orthorhombic phase is mainly distributed within the range from 70 to 90° in Fig. 4(b). However, as shown in Fig. the P-V loop is irregular and distorted because the HfO_2_ is located into the microcavities, which results that the electrode partly contact with the chemically-etched surface of Si. Though interpretations have been extensively discussed and debated for the ferroelectricity of HfO_2_ in recent years. The presence of ferroelectric shape of the P-V loop and XRD spectra for PS with HfO_2_ filled into its microcavities, could still imply the presence of ferroelectricity in this work. The incorporation and encapsulation of Si could promote the ferroelectric phase transformation^27^. Though the mixture of HfO_2_ with Si in the nanometer microcavities shown in this work is not entirely the same with the directly Si insertion into HfO_2_, The similar influence between them for the adjustment of ferroelectricity of HfO_2_ could be expected.

In Fig. 2, there are three PL subpeaks obviously present within the broad blue emission, for each sample annealing at different temperatures. It is ascribed to the recombination from defect states to valance band (E_V_) of HfO_2_, for the  and  subpeaks located at 375 nm (3.3 eV) and 430 nm (3.0 eV), respectively (except for the blue subpeak of  which is from porous Si). The  and  subpeaks could be from the energy transition of defects levels in HfO_2_, because the energy of band-to-band recombination of HfO_2_ (5.9 eV) is too much higher even than that of the 375 nm irradiation^29^,^30^,^31^,^32^. Since the HfO_2_ dielectric fabricated by sputtering was commonly in oxygen-deficient state^26^,^33^,^34^, the defects levels were probably originated from oxygen vacancies. This was confirmed by the control annealing in oxygen atmosphere as shown in Fig. 5(a), since the intensities of the  and , both decrease with increasing of the annealing temperatures in oxygen ambient. Increasing the annealing temperature in oxygen reduces the oxygen vacancy concentration in the HfO_2_ dielectric, therefore, it is reasonable that oxygen vacancies should be the dominant source for the defect states. Meanwhile, the corresponding red subpeaks,  and , are also reduced for the effectively reduction of oxygen vacancies by annealing in oxygen, as shown in the Fig. 5(b), which implies that the  and  are ascribed to the emission from HfO_2_ dielectric. The annealing in vacuum enhances these emissions as shown in Fig. 5, which could be attributed to the increase of oxygen vacancies for the oxygen escape and the oxygen adsorb ability of Si from HfO_2_. Above all, photogeneration of carriers not only occur in Si crystals, but also can take place in HfO_2_ layer. Via this way, carriers for recombination are greatly increased. HfO_2_ may not only confine carriers but also contribute more carriers for recombination.

RETRACTED

The blue subpeaks from HfO_2_, i.e.,  and , are located at 3.3 eV (375 nm) and 3.0 eV (430 nm), respectively. Correspondingly, the red subpeaks from HfO_2_, i.e.,  and , are located at 1.7 eV (750 nm) and 1.4 eV (860 nm), respectively. The above results are consistent with the previous reports that the PL bands of HfO_2_ are located at 1.4–1.8 eV (690–890 nm) and at 2.1–3.5 eV (354–590 nm)^29^,^32^,^35^. We have checked the strongest excitation energy during PL measurement, it is found that 4.7 eV is most favaroubale, which should correspond to the dominating defects lies at 4.7 eV above the valence band. Therefore, it could be reasonable that the irradiation in HfO_2_ dielectric was probably from the band-to-band transition due to the oxygen vacancy defect levels. The transition process may as below: The carrier first is excited to the defect states of 4.7 eV above E_V_ and then relaxed to the defect states of 3.3 and 3.0 eV, with the energy difference of 1.7 and 1.4 eV which corresponding to the red emission  and . Then, the relaxed carriers were recombined in the valence band with a luminance with the blue emission 3.3 and 3.0 eV, which are consistent with the blue subpeaks of  and , respectively. The energy level of the defect states are schematically shown in Fig. 6.

Additionally, the annealing temperature dependence of the integrated blue PL intensity was shown in Fig. 7. In most light-emission systems^36^,^37^, PL quenches very strongly with increasing annealing temperature at the high temperature, making heat treatment problematic in luminescence device applications. However, in our films it was observed that the PL intensity increased as annealing temperature increasing for both low and high temperature (high up to 900 °C). Therefore, the device is partly free from the disturbance of the temperature quenching effect in the annealing process. Strong temperature quenching of PL at high temperature is generally a result of the strong temperature dependence of competing non-radiative routes, which could be attributed to the thermally activated crossover from the excited state to the ground state, multiphonon relaxation, and thermally activated photoionization — while the band-to-band transition is relatively temperature-independent^38^. Here, spatial localization of the radiative carrier population decouples it from any non-radiative recombination occurring elsewhere, thus eliminating luminescence quenching.

RETRACTED

In summary, HfO_2_ was deposited by low power sputtering into the microcavities of Si, enhancement of the blue PL peak was observed. In PL spectra, the broad band light was emitted from both the HfO_2_ dielectric and the porous Si. The blue emission from Si could be enhanced by the ferroelectricity of HfO_2_. HfO_2_ not only confines the diffusion of carriers due to its polarized field but also contributes more carriers for recombination. The observation of visible blue light emission of Si filled with HfO_2_ dielectric is remarkable as both HfO_2_ and Si are highly compatible with Si-based electronic industry.

## Additional Information

**How to cite this article**: Jiang, R. *et al.* Enhancement of the blue photoluminescence intensity for the porous silicon with HfO_2_ filling into microcavities. *Sci. Rep.* **5**, 15574; doi: 10.1038/srep15574 (2015).

## Figures and Tables

**Figure 1:** Flow-process illustration for the HfO_2_ filled porous Si with microcavities.

**Figure 2:** Typical PL spectra for the samples with HfO_2_ filled into the Si microcavities. B and R, denotes the blue subpeak and red subpeak, respectively. The top number (1, 2 and 3) is the order of subpeaks. The bottom symbol of “Si” and “HfO_2_” is the origination of emission. The samples were annealed in vacuum at 500, 700 and 900 °C, respectively. For comparison, the PL spectrum of as-deposited sample was also shown. Inset is the images of blue light emission for samples annealed at 500, 700 and 900 °C, respectively.

**Figure 3:** Cross-sectional SEM image of (a) cross section of the porous silicon without HfO_2_ filling and (b) with HfO_2_ filling. (**c**) is the frontside SEM image of the porous silicon layer. (**d**) is the Hf 4*f* core level spectra for HfO_2_-filling samples. Silicide subpeaks can be observed for samples, which implies the introduction of Si within HfO_2_ dielectric. From deconvolution, it consists of Hf-Si bond (Hf 4*f* 5/2 :18.9 eV; Hf 4*f *7/2 :17.4 eV) besides Hf-O component (Hf4*f* 5/2 :18.5 eV; Hf 4*f* 7/2 :16.8 eV). The diagram of microcavities filled with HfO_2_ in porous Si is shown in the inset.

RETRACTED

**Figure 4:** (**a**) P-V hysteresis measurements of the HfO_2_ filled into microcavities of porous silicon at 900 °C. (**b**) GIXRD data for a series of samples annealing at 500, 600 and 700 °C, respectively. The inset shows the standard peak position for the monoclinic, orthorhombic, tetragonal and cubic phase structure, which were used for the comparison.

**Figure 5:** The intensities of luminescence from HfO_2_ vs. the annealing temperatures. (**a**) The blue subpeaks, i.e.,  and , annealing in vacuum and oxygen, respectively. (**b**) the red subpeaks, i.e.,  and , annealing in vacuum and oxygen, respectively.

**Figure 6:** Schematic diagram for the light emission from HfO_2_ by the transitions in the energy levels of defect states.

**Figure 7:** Integrated blue PL intensity as a function of the annealing temperature in vacuum.
